The article "Dispersal Routes and Habitat Utilization of Juvenile Atlantic Bluefin Tuna, Thunnus thynnus, Tracked with Mini PSAT and Archival Tags" was published in 2012. Journal: PLoS One.

# Dispersal Routes and Habitat Utilization of Juvenile Atlantic Bluefin Tuna, *Thunnus thynnus*, Tracked with Mini PSAT and Archival Tags

**DOI:** 10.1371/journal.pone.0037829

**Published:** 2012-05-22

**Authors:** Benjamin Galuardi, Molly Lutcavage

**Affiliations:** Large Pelagics Research Center, University of Massachusetts Amherst, Gloucester, Massachusetts, United States of America; National Oceanic and Atmospheric Administration/National Marine Fisheries Service/Southwest Fisheries Science Center, United States of America

## Abstract

Between 2005 and 2009, we deployed 58 miniature pop-up satellite archival tags (PSAT) and 132 implanted archival tags on juvenile Atlantic bluefin tuna (age 2–5) in the northwest Atlantic Ocean. Data returned from these efforts (n = 26 PSATs, 1 archival tag) revealed their dispersal routes, horizontal and vertical movements and habitat utilization. All of the tagged bluefin tuna remained in the northwest Atlantic for the duration observed, and in summer months exhibited core-use of coastal seas extending from Maryland to Cape Cod, MA, (USA) out to the shelf break. Their winter distributions were more spatially disaggregated, ranging south to the South Atlantic Bight, northern Bahamas and Gulf Stream. Vertical habitat patterns showed that juvenile bluefin tuna mainly occupied shallow depths (mean  = 5–12 m, sd  = 15–23.7 m) and relatively warm water masses in summer (mean  = 17.9–20.9°C, sd  = 4.2–2.6°C) and had deeper and more variable depth patterns in winter (mean  = 41–58 m, sd  = 48.9–62.2 m). Our tagging results reveal annual dispersal patterns, behavior and oceanographic associations of juvenile Atlantic bluefin tuna that were only surmised in earlier studies. Fishery independent profiling from electronic tagging also provide spatially and temporally explicit information for evaluating dispersals rates, population structure and fisheries catch patterns.

## Introduction

Management of Atlantic bluefin tuna (*Thunnus thynnus*) is shared by the International Commission for the Conservation of Atlantic Tunas (ICCAT) and national fisheries management agencies. In recent years, new information on migration patterns for adult western Atlantic bluefin tuna (ABFT) has revealed even stronger habitat connectivity among distant oceanic regions [1]–[3] than indicated by fisheries patterns and conventional tagging [4]–[6]. Between April and October, an extensive recreational fishery exists for juvenile ABFT off the U.S. coast from Maine to North Carolina (approximately 35°–44°N, and 68°–75°W). Recent studies showed over 50-% of juvenile fish sampled for biochemical markers were assigned a Mediterranean origin [2], [7], highlighting the need for further study into trans-Atlantic movements and mixing. Determination of the spatial structure and life history of the ABFT population relies on knowledge of juvenile dispersal patterns and year-round habitat utilization, and remains an important goal for stock assessment [8].

The article "Dispersal Routes and Habitat Utilization of Juvenile Atlantic Bluefin Tuna, Thunnus thynnus, Tracked with Mini PSAT and Archival Tags" was published in 2012. Journal: PLoS One.

While adult bluefin tuna are exploited in the commercial fishery in the western Atlantic, juveniles are highly sought by recreational anglers, and constitute a multi-million dollar sport fishery. Conventional tagging and fisheries catch patterns have revealed dispersal patterns of juvenile ABFT in West Atlantic coastal areas during summer and fall [6], [9], [10] but their winter and springtime movements and behavior have only been surmised. Fisheries expeditions in the 1950's and ‘60s found that some juvenile ABFT occupied the Gulf Stream over winter [6], [11], but no exploratory cruises have taken place since then.

Since 1999, pop-up satellite archival tags (PSATs) applied to adult ABFT have produced a large body of information on their movements and habits [3], [12], [13] but until recently, PSAT tags were too large to be applied to small individuals. In 2005, we began the Tag-a-Tiny ™ program, a multiyear project to study juvenile ABFT life history, utilizing conventional and electronic tags (in collaboration with AZTI Technalia, Gipuzkoa, Spain). In 2007, following commercial development of a mini-PSAT, (X-tag, Microwave Telemetry, Inc) we expanded the study and deployed mini PSATS on juvenile ABFT in the Gulf of Maine between 2007 and 2009.

## Methods

### Implanted Archival Tags

Between 2005 and 2008 we tagged 132 Atlantic bluefin tuna with implanted archival tags. Fishing and tagging work was conducted from charter or commercial fishing vessels out of the ports of Wachapreague, VA, Gloucester, MA, and Chatham, MA (USA). All fish were captured by rod and reel using J-hooks. Tagged fish sizes were 66–145 cm curved fork length (CFL, mean±sd; 86.5±14 cm, Fig. 1). Tag models were Wildlife Computers MK-9 (n = 20), Lotek LTD 2310 (n = 82) and LTD 2350 (n = 30) (Table 1). We used previously developed tag implant methods [14]–[16] following standard veterinary practice. Briefly, once fish were hooked, we brought them aboard using a vinyl stretcher, placed a dark wet cloth over their eyes, and determined their condition. Suitable individuals were placed ventral side up in a custom built tagging cradle and measured. A small incision was made to create access to the intraperitoneal (IP) cavity, and the archival tag was inserted into the cavity. The incision was closed with two sutures and Vetbond was applied to seal the incision. We also applied a conventional ID tag near the base of the second dorsal fin notifying finders of the implanted archival tag. The entire procedure usually took less than 90 sec to complete and the fish was then released. Fish tagged with Wildlife Computers tags followed a dorsal musculature implant procedure [16]. This was discontinued due to the slightly larger size of the LTD 2310 tags and to be consistent with other successful tagging programs efforts utilizing IP implants on small tunas [*e.g*. 17, 18–21]. All archival tags were programmed to record internal and external temperature, light, and pressure (depth) once per minute. This rate of measurement was estimated to support 3–5 years of data storage for these tag models.

The article "Dispersal Routes and Habitat Utilization of Juvenile Atlantic Bluefin Tuna, Thunnus thynnus, Tracked with Mini PSAT and Archival Tags" was published in 2012. Journal: PLoS One.

**Figure 1:** Length distribution of juvenile bluefin tuna tagged with implanted archival tags (white boxes) and X-tags (grey boxes), 2005–2009. A total of three years classes are present although a single year class (the 2003 cohort; age 2 in 2005) was clearly dominant (note the yearly increase in size of tagged fish).

**Table 1:** Summary of implanted archival tagging efforts in Eastern Virginia and the Gulf of Maine, 2005–2008.

	E. Virginia	Gulf of Maine	Total
**WC MK-9**			
**2005**	20		20
**LTD 2310**			
**2005**	26	52	78
**2006**	4		4
**LTD 2350**			
**2006**	10	13	23
**2007**		5	5
**2008**		2	2
**Total**	**60**	**72**	**132**

The left column indicates manufacturer (WC and LTD denote Wildlife Computers and Lotek respectively) and model number.

### PSAT tagging

We deployed mini PSATs (X-tags) in August – October 2007 (n = 32), 2008 (n = 22) and 2009 (n = 4) on ABFT (105–168 cm CFL, Fig. 1) off Cape Cod (Massachusetts, USA, Table 1). All tagging was conducted aboard the fishing vessels by rod and reel. Fish were brought on board and a wet towel placed over the eyes and measured for curved fork length (CFL) and finlet samples were taken for further genetic analysis and determination of natal origin. Tag and tether assemblies, materials and tagging procedures were similar to those previously described for adult ABFT [13], [22], with tether length adjusted for smaller fish. Tags were attached by inserting the dart near the base of the second dorsal fin. In 2007, we experimented with a secondary attachment to reduce tag movement during swimming (n = 16). This consisted of a short length of monofilament in a crimped loop, attached to a small white nylon dart. T-tests indicated this did not make a significant difference in attachment duration (days attached with tether, x = 197 days, no tether, x = 201 days, p = 0.9477), and the practice was discontinued in subsequent years. We performed all field work under National Oceanic and Atmospheric Administration exempted fishing permits TUNA-EFP-07-01, TUNA-EFP-08-03, TUNA-EFP-09-03 for years 2007, 2008 and 2009, respectively.

The article "Dispersal Routes and Habitat Utilization of Juvenile Atlantic Bluefin Tuna, Thunnus thynnus, Tracked with Mini PSAT and Archival Tags" was published in 2012. Journal: PLoS One.

**Table 2:** Tagging Summary for 26 juvenile Atlantic bluefin tuna tagged with X – tags which returned data (out of 58) and one recovered implanted archival tag (*).

Tag ID	Tagging Date	CFL (cm)	Tag latitude N	Tag longitude W	Report Date	Report latitude N	Report longitude W	Days at Liberty
2005-B5082*	9/9/2005	79	41.457	69.299	8/31/2010	NA	NA	1817
2007-34457	8/13/2007	130	41.632	69.530	8/23/2007	41.892	69.268	10/365
2007-36973	8/13/2007	124	41.629	69.543	8/17/2007	41.944	69.318	4/365
2007-36169	8/13/2007	121	41.621	69.549	2/12/2008	34.867	75.817	183/365
2007-36159	8/13/2007	168	41.584	69.563	1/27/2008	38.712	59.746	167/365
2007-36154	8/20/2007	117	41.557	69.607	8/24/2007	41.850	69.341	4/365
2007-34458	8/20/2007	105	41.572	69.559	10/4/2007	41.028	70.375	45/365
2007-34459	8/20/2007	119	41.568	69.536	9/17/2007	41.804	69.545	28/365
2007-36557	8/27/2007	124	41.577	69.604	8/27/2008	38.470	74.194	366/365
2007-36086	8/27/2007	122	41.462	69.354	8/27/2008	41.643	69.559	366/365
2007-36203	8/27/2007	122	41.445	69.373	8/27/2008	37.376	72.915	366/365
2007-36091	8/27/2007	123	41.448	69.380	1/28/2008	39.768	69.362	154/365
2007-36210	8/27/2007	124	41.455	69.364	8/27/2008	41.462	69.111	366/365
2007-36092	9/5/2007	124	41.489	69.387	10/1/2007	40.373	72.245	26/365
2007-36093	9/5/2007	122	41.457	69.373	2/25/2008	34.679	75.636	173/365
2007-36090	9/5/2007	124	41.415	69.355	9/5/2008	41.801	69.411	366/365
2007-36208	9/5/2007	124	41.404	69.351	6/23/2008	38.310	74.643	292/365
2007-36041	9/5/2007	130	41.405	69.366	9/5/2008	42.102	70.241	366/365
2007-36205	9/5/2007	117	41.395	69.374	1/4/2008	34.868	75.360	121/365
2007-36638	9/5/2007	122	41.394	69.345	6/26/2008	36.933	74.902	295/365
2007-36204	9/11/2007	119	42.082	70.266	9/11/2008	41.803	69.136	366/365
2007-36088	10/2/2007	125	41.428	69.373	1/19/2008	35.239	75.049	109/365
2008-82977	6/27/2008	139	41.605	69.566	6/27/2009	42.157	70.193	365/365
2008-82986	10/8/2008	145	41.487	69.376	9/18/2009	41.745	69.820	345/365
2009-95161	9/21/2009	115	41.667	69.867	5/15/2010	36.423	75.600	236/236
2009-95160	9/21/2009	132	41.667	69.783	5/15/2010	39.106	68.458	236/236
2009-95167	9/21/2009	116	41.800	69.867	5/15/2010	39.504	69.601	236/236

Only tags which returned data are present. The recovered implanted archival tag was caught in Cape Cod Bay, Massachusetts. Exact coordinates were not available nor relevant to analysis.

The mini PSATs used in this study were programmed to release after 12 months and to record external temperature and pressure (depth) every 15 minutes. All tags had a failsafe release set at 4 days, which would indicate post-release mortality or premature tag release. As the tags continued to be developed and improved during this study, the manufacturer changed several programming settings. In 2007, X-tags capabilities mirrored that of the manufacturer's standard size PTT-100 tag. This is described in detail elsewhere [22] and on the manufacturer's website (www.microwavetelemetry.com). X-tags deployed after 2007 recorded light, external temperature (0.01 C°) and depth (0.33 m) every two minutes in a separate part of the memory, accessible if the tag is recovered. Additionally, X-tags manufactured after 2007 have a variable depth measurement precision as follows: readings above 86 m  = 0.67 m, 258–86 m  = 1.34 m, 602–258 m  = 2.69 m and 602–129 1m  = 5.38 [23]. The differences resulted from an increase from 8-bit to 12 bit memory, allowing more divisions between the minimum and maximum depth (i.e. 256 divisions for 8-bit memory and ∼1377 m maximum depth yields 5.38 m accuracy). This was a major improvement over the standard 5.38 m resolution possible in tags deployed through 2007. While the PTT-100 has diode placement allowing 360 degrees of light sensing in the nosecone, the X-tags light sensor was located in the body of the tag.

The article "Dispersal Routes and Habitat Utilization of Juvenile Atlantic Bluefin Tuna, Thunnus thynnus, Tracked with Mini PSAT and Archival Tags" was published in 2012. Journal: PLoS One.

**Figure 2:** Reference map of study area (panel A) and all reconstructed tracks from 2007 –2009 X-tagged juvenile bluefin tuna (n = 26). The period of July 2007 through September 2010 is represented. Panel B) shows tagged fish by year tagged while panel C) shows utilization distribution (UD) aggregated for all tagged fish during their time at liberty. The overall distribution indicates core-use areas off Cape Cod, Long Island and the mid-Atlantic coast. The color terminates at the 95% UD (side-use area).

**Figure 3:** Utilization distributions aggregated for all PSAT tagged juvenile Atlantic bluefin tuna for each month. Core-use areas are spatially constrained in summer months (July–Sept.) and are more dispersed in winter months (Jan. – March). Fall months show a southern migration along the shelf break and increase in spatial dispersal while spring months show the reverse trend.

### Horizontal movement

For juvenile ABFT tagged with X-tags we first discarded spurious measurements by setting upper and lower limits on where the fish might have traveled (20°N, 50°N, 100°W and 20°W). We then used a state space unscented Kalman filter with blended sea surface temperature [24]. The sea surface temperature (SST) product chosen for this analysis was an 11 km, 8-day composite product comprised of several far-infrared and microwave SST products (MODIS, AVHRR, GOES, AMSR-E: NOAA CoastWatch Program, NOAA NESDIS Office of Satellite Data Processing and Distribution, and NASA's Goddard Space Flight Center, OceanColor Web). SST's experienced by each fish were defined as the maximum temperature recorded for a given day. SST values for days where temperature was not observed were interpolated using local polynomial smoothing [25] utilizing the surrounding day's maximum temperatures. Following UKFSST position estimation, we used a secondary bathymetric correction [3], [25] which rejected days where suitable bathymetry values could not be extracted from within the confidence interval estimated in the UKFSST step. Days with missing positions, and their uncertainty, were then interpolated using loess smoothing and linear interpolation [26], respectively, and corrected for bathymetry. In this fashion, we estimated daily positions for the entire duration at liberty with no missing days. These processes were compiled in the analyzepsat library for R [27]. The recovered archival tag recorded external and internal temperature, light, and pressure once per minute. As light curves are readily available, horizontal paths may be reconstructed from archival tags using a variety of techniques [28]–[30]; here we used UKFSST, with blended SST, followed by bathymetric correction.

The article "Dispersal Routes and Habitat Utilization of Juvenile Atlantic Bluefin Tuna, Thunnus thynnus, Tracked with Mini PSAT and Archival Tags" was published in 2012. Journal: PLoS One.

**Figure 4:** Total utilization distribution area for 26 PSAT tagged juvenile Atlantic bluefin tuna aggregated by month. The 50% line shows the fluctuation in core-use areas while the 95% line shows the dramatic seasonal shifts in wide-use areas.

**Figure 5:** Aggregated diel depth (A) and temperature (B) records for 26 juvenile Atlantic bluefin tuna at liberty for up to one year. There are no overall diel differences in either depth or temperature. The temperature graph shows a bimodal temperature distribution indicative of differences in summer and winter habitat. The depth plot shows that JBFT spend more than 70% of their time in depths 30 m or shallower.

**Figure 6:** Diel temperature A) and depth B) differences by month for 26 PSAT tagged juvenile Atlantic bluefin tuna. Boxplots (white  =  day, grey  =  night) show mean and interquartile range. There were no seasonal differences in diel depth and temperature in any month, but variation in temperature was greater in winter months than in summer months. Vertical habitat compression is prominent in summer months while vertical habitat expansion exists in winter months.

### Utilization areas

Areas of core activity of X-tagged bluefin tuna were determined directly from the uncertainty bounds of all fish across years [3], [31]. Gridded probability density was calculated per 0.1° cell covering the entire range (20°N, 50°N, 100°W and 20°W) and converted to a volume. These were used to generate overall and monthly utilization distributions to determine high use areas throughout the year, using the adehabitat package for R [32] as well as custom functions included in the analyzepsat package.

The article "Dispersal Routes and Habitat Utilization of Juvenile Atlantic Bluefin Tuna, Thunnus thynnus, Tracked with Mini PSAT and Archival Tags" was published in 2012. Journal: PLoS One.

### Vertical habitat envelopes

We determined vertical habitat utilization via construction of vertical habitat envelopes [33], [34] which were determined by month across all tagging years for all fish with days at liberty >20 days (n = 23). Since X-tags used in this study had varying depth sensitivities, we standardized across years by binning depths into 5 m groups and 1°C increments. Depths greater than 250 m were a single bin given their low frequency. Log frequency counts were then made for each temperature depth combination.

Depth and temperature data from X-tags is transmitted as a delta value from a reference measurement. These measurements occur every 15 minutes at midnight (0:00), 06:00, 12:00 (noon), and 18:00 GMT. Subsequent measurements are stored as delta values from the previous hour's value (i.e., 07:15 is the difference from 06:15). This limits the maximum change which may be transmitted through data packets sent to the Argos satellite. This is most noticeable in a deep, rapidly diving animal such as a bluefin tuna and in practical terms, means that depth changes +/−86 m from the previous hour's value are not reliable [23]. For this reason we removed all depth values not taken at the reference times and >86 m change from the previous hours measurement. This resulted in removal of 1.2% of all depth data.

**Figure 7:** Vertical habitat envelopes for 26 PSAT tagged juvenile Atlantic bluefin tuna. Depths were binned at 5 m increments and include a bin for all values deeper than 250 m. Temperatures were binned at 1°C. The scale indicates log of the frequency (counts) for each temperature depth combination for all PSAT tagged JBFT monthly. Winter envelopes indicate a bi-modal temperature and depth distribution reflective of the spatial range expansion and the varying oceanic regimes inhabited. Summer envelopes are more concentrated in temperature and depth indicative of the spatial range contraction to more homogeneous water masses on the continental shelf and at the shelf break off the northeast U.S.

**Figure 8:** Recovered implanted archival tag showing external temperature (A, C, and E) and corresponding reconstructed migration (B, D and F) referenced by season. Colored bars in panels A, C and E correspond to the season color on the corresponding maps (panels B, D and F). Clear seasonal differences can be seen through the 30 months data were collected. When the fish inhabited well mixed water the depth patterns were more variable, with deep excursions and deeper mean depths. In summer months, in well stratified water, this fish had a more shallow depth distribution.

The article "Dispersal Routes and Habitat Utilization of Juvenile Atlantic Bluefin Tuna, Thunnus thynnus, Tracked with Mini PSAT and Archival Tags" was published in 2012. Journal: PLoS One.

**Figure 9:** An 8-day blended SST composite (AVHRR, MODIS, AMSR-E and GOES) centered on March 31, 2008 and corresponding locations from tagged JBFT at that time (n = 9). The black line marks the 20°C contour and shows a rough outline of the Gulf Stream at this time of year. This figure illustrates juvenile Atlantic bluefin tuna spatial disaggregation in winter months as well as the importance of the Gulf Stream as a winter habitat.

## Results

We recovered X-tag data from 26 Atlantic bluefin tuna producing records from 4 days to one year (215±137 days). These included five tag records <30 days and nine tag records >300 days (Table 2) X-tags have a constant pressure release mechanism which indicates when a tag is resting at the bottom and, in the case of a tuna, can be indicative of mortality. All reporting tags were either shed early for unknown reasons or reported on time and depth patterns showed no evidence of post release mortality. There was a large disparity in reporting rates between tagging years: 2007, n = 21/32, 2008, n = 2/22, 2009, n = 3/4. The high non-reporting rate for 2008 deployments was attributed by the manufacturer to a software problem present in tag batches that year (Dr. Paul Howey, Microwave Telemetry, Inc, personal communication).

Size distributions of tagged fish included three distinct modes, dominated by a strong 2003 year class (Fig. 1). Our combined archival and PSAT tagging efforts track the growth of the 2003 year class and represent a consistent tagging effort through four years of this cohort. According to published growth curves for ABFT [35], we incrementally tagged primarily 2–5 year old fish from the 2003 year class in 2005 to 2008, respectively. Across all years of tagging we also tagged individuals in the 2002 (n = 4) and 2004 (n = 5) year classes (see outliers in Fig. 1).

Fish tagged with X-tags occupied the continental shelf and Gulf Stream margin from the Gulf of Maine to the South Atlantic Bight. One fish each in 2007 and 2009 travelled into the central north Atlantic (Fig. 2a). Two fish tagged in 2008 moved farther south (to the northern Bahamas) than those tagged in other years. Overall, core habitat utilization areas emerged southeast of Cape Cod (MA), south of Long Island, and at the shelf break from the Eastern Shore of Virginia to Cape Hatteras (Fig. 2b). Robust recreational fisheries exist for juvenile ABFT in these areas, as well as off the coast of New Jersey, USA. Although we had small sample sizes in two tagging years, overall patterns were not different between years (Fig. 2a). Notably, the largest fish in our study, tagged in 2008, displayed the most extensive southern range.

The article "Dispersal Routes and Habitat Utilization of Juvenile Atlantic Bluefin Tuna, Thunnus thynnus, Tracked with Mini PSAT and Archival Tags" was published in 2012. Journal: PLoS One.

Spatial distribution of juvenile ABFT varied seasonally both in core location and extent of distribution (Fig. 3). Summer (July – Sept.) distributions were more restricted to coastal areas; the Gulf Stream margin and shelf break north of Cape Hatteras, extending to the southern Gulf of Maine. In autumn, (Oct. – Dec.) a transitional period, core use areas shifted southward. By December, no tagged fish remained in the Gulf of Maine, and 50% utilization distributions were centered off the Eastern Shore of Virginia to Cape Hatteras. Winter (Jan. – March) spatial distributions were the largest in area and ranged farther south than in other seasons. In spring (April – June) tagged fish returned to areas north and west, constricting their overall range. In April, core-use areas were centered off Cape Hatteras, North Carolina. ABFT that retained their tags for the full year either returned to the Gulf of Maine (n = 5) or were off the coast of New Jersey (n = 2) when the tags reported.

Area occupied at the 95% utilization level (wide-use area) reached a maximum of over 10,000 km^2^ during February – April, while in September the 95% area was only 1,775 km^2^ (Fig. 4). Core-use (50%) areas during February – April were 1,209, 1,277 and 1,180 km^2^, respectively, while the September area was 362 km^2^. This illustrates ∼66% contraction in home range between winter and summer peaks, while wide-use areas contracted by an order of magnitude for the same periods.

### Vertical activity and temperature

Although the maximum recorded depth for PSAT tagged fish was 800 m, they spent the majority of time at relatively shallow depth (<20 m, Fig. 5). There was no diel difference in the overall distribution of depths and temperatures. Depth and temperature data was pooled by month across year to examine seasonal differences. Juvenile ABFT experienced a wide range of sea temperatures (4–26°C) and showed seasonal patterns of temperature preference and variability. The warmest months were June – September where mean sea temperature was 17.9–20.9°C, also when the standard deviation of thermal profiles decreased from 4.2°C in June to 2.6°C in September. Mean depths during the summer were between 5 and 12 m with standard deviation 23.7 m decreasing to 15 m in June – Sept., coincident with the temperature decrease. In contrast, during January-May, mean depth associations were 41–58 m with larger standard deviations (48.9–62.2 m). No diel differences were apparent in any month (Fig. 6).

Vertical habitat utilization envelopes constructed for juvenile ABFT showed distinct seasonal habitat differences. In winter (Jan. – March), two core use areas appear centered around 100 m and ∼40 m, with habitat centered at 12°C and 21°C, respectively (Fig. 7). In summer (July –September) tagged fish displayed a sharp compression in vertical habitat, with core areas near the surface and temperatures centered around 15–20°C. Spring and fall habitat indicated transition in depth regime between a bimodal, deeper winter distribution and shallow summer regime. By winter, there is a distinct shallow (0–30 m) and relatively cool (9–13°C) core distribution in November and by December, a general deepening of vertical habitat and two modes of core use temperature are evident.

The article "Dispersal Routes and Habitat Utilization of Juvenile Atlantic Bluefin Tuna, Thunnus thynnus, Tracked with Mini PSAT and Archival Tags" was published in 2012. Journal: PLoS One.

In winter, juvenile ABFT had a bimodal distribution, and were widely distributed across sub-tropical (i.e., warm winter temperatures) and temperate (cooler) oceanic conditions (Fig. 3). In summer, their vertical habitat was associated with strong, shallow thermoclines in the Gulf of Maine and mid-Atlantic shelf areas.

### Archival tagged fish

In September, 2010, we recovered an implanted archival tag (B5082, Lotek) from a fish recaptured in Cape Cod Bay, MA that had been at liberty for five years. Although there were three validated recaptures where fish were subsequently released alive, this represents the only recovery to date from the 132 fish tagged. The recovered tag yielded 30 months of data, over 2.6 y, but less than mission life estimated by the manufacturer. This fish was 79 cm CFL at release and 180 cm CFL at recovery, for a mean annual growth rate of 20 cm.

The reconstructed horizontal track indicated that the tagged fish remained on shelf break with occasional forays off the shelf into the Gulf Stream and South Atlantic Bight. (Fig 8, panels b, c and f). Initially, the fish remained in the Gulf of Maine until mid-October, and then moved south to the Mid-Atlantic Bight. This individual stayed in a narrow longitudinal band along the mid-Atlantic shelf region throughout 2006, the only exception being a brief excursion south in March into subtropical water near 29°N and 72°W. In 2007 the fish traveled along a wider longitudinal range and twice returned to the Gulf of Maine, in summer (July) and late autumn (Oct–Nov., 2007) before heading south again. The tagged stopped recording in February 2008 when the fish occupied the Gulf Stream recirculation area, the most northern winter location observed for this individual.

The returned tag provided a detailed (i.e., one minute) record of its oceanographic regime (Fig. 8a, 8c, and 8e). Maximum recorded depths were in excess of 800 m, usually during winter (Jan. – March). Mean depths in summer were between 10–20 m and increased in autumn to 40–60 m, with seasonal cooling, when the fish moved southward. The largest variability in depth occurred in winter when frequent deep excursions were observed. From June 2006 through February, 2007, this fish ranged between Cape Hatteras and the shelf break south of Long Island (Fig 8b and 8d). Changing oceanographic conditions are visible in external temperature records (Fig. 8a and 8c). This fish did not visit the Gulf of Maine in 2006, but in 2007 entered the Gulf of Maine twice, in June and October (Fig. 8e and 8f). Overall, including recapture, this individual entered the Gulf of Maine a minimum of four times, consistent with the seasonal site fidelity observed in PSAT-tagged ABFT in this study. In 2007, the data record also places this individual in the same seasonal core use areas as individuals tagged with PSATs.

The article "Dispersal Routes and Habitat Utilization of Juvenile Atlantic Bluefin Tuna, Thunnus thynnus, Tracked with Mini PSAT and Archival Tags" was published in 2012. Journal: PLoS One.

## Discussion

This study provides the first fishery-independent information on year-round spatial and vertical distribution of juvenile bluefin tuna in the northwest Atlantic and provides extensive data describing their year-long dispersal patterns and habitat utilization. The Gulf Stream emerged as an important juvenile habitat from autumn through spring (Fig 9). While core use areas centered mostly on the shelf margin, winter and spring distributions in the South Atlantic Bight are coincident with Gulf Stream position [*e.g*. 36]. Unfortunately, the low rate of recovery of implanted archival tags and low reporting rate from our 2008 X-tags prohibited a robust length-based comparison of habitat use. This study provides fishery independent confirmation of exploratory cruise and commercial fisheries observations of the 1950's–1970's [6], [11] establishing the importance of the Gulf Stream region while providing greater details on seasonality and range of other habitats of juvenile ABFT.

Although not designed as a post-release mortality study *per se*, tag records show no evidence of mortality over observation periods of up to one year. All fish were caught on J hooks via rod and reel using conventional recreational fishing techniques (*e.g*., cedar plugs, squid rigs). The high survivorship is consistent with our tagging results for giant bluefin tuna [3], [13], [22] and juveniles tracked up to 48 h with sonic tags [37], and suggests that if properly handled, juvenile ABFT are hardy, and an appropriate species for tag and release programs.

Maximum depths achieved by juvenile ABFT in this study were consistent with tag records from age 2 fish studied in the Mediterranean [18] and in the Bay of Biscay (Dr. Nicholas Goñi, pers. comm.). Spatial distribution in summer months was also generally consistent with the timing and locations of the U.S. recreational bluefin fishery. Although we tracked 14 juvenile ABFT for at least 8 months, it is notable that we did not observe trans-Atlantic migrations.

The article "Dispersal Routes and Habitat Utilization of Juvenile Atlantic Bluefin Tuna, Thunnus thynnus, Tracked with Mini PSAT and Archival Tags" was published in 2012. Journal: PLoS One.

Archival tagging of smaller (<100 cm) juvenile ABFT in the Mediterranean Sea [18], demonstrated similar physiological capabilities in terms of their thermal profiles and maximum depth achieved (765 m). In both studies, despite size differences, fish displayed similar seasonal changes in depth patterns, such as surface oriented activity in summer months, with few excursions below 200 m (150 m is noted in Yamashita and Miyabe, 2001). Depth and temperature patterns also exhibited distinct regime shifts, corresponding to fish traveling to, and residing in different ocean water masses, where they presumably targeted different prey. Similarly, juvenile Pacific bluefin tuna tagged off the Japanese coast had different vertical behavior in the East China Sea and the Kuroshio-Oyashio transition region, attributed to the depth of anchovy biomass [38] highlighting the strong behavioral link between predator and prey in bluefin distribution. Bluefin tuna warm their retinas, enhancing vision, and unique anatomical and physiological adaptations conferring endothermy [39], [40] make them highly efficient predators. A visceral rete warms their stomach [41] and highly efficient digestive enzymes support rapid digestion of prey [42], [43]. Thermal (4–26°C) and depth profiles (to 800 m) of juvenile ABFT suggest they hunt prey to their maximum depths attained, and despite smaller body size, approach those documented in much larger, adult fish, *e.g*.,3–30°C, 0– >1000 m, [44], [45].

In sonic tracking studies, small (74–106 cm CFL) ABFT tracked with their schools off the Eastern Shore of Virginia [37] dove regularly to the seabed while feeding on sandlance (*Ammodytes* sp), their preferred prey in the mid-Atlantic and New England region [10], [46], [47] Recent diet studies suggest that ABFT experience ontogenetic shifts in diet of several trophic levels from age 1–2 to adulthood [47]. Although our sample size is small, comparing the largest (Fig. 2, 2008 tagged fish) and smallest (archival tag) fish in our study suggests that horizontal range expansion most likely occurs with as fish increase in size. This could indicate greater energetic capability to search for prey beyond easily accessible, but perhaps less energy-rich forage grounds, [48], [49] but this is not easily resolved with conventional diet analysis and current tag technologies. In comparison with juvenile yellowfin and bigeye tunas [50]–[52], juvenile ABFT display greater plasticity and range in habitat and presumed sensory and thermal capabilities, which supports their fast growth and unique life history.

The article "Dispersal Routes and Habitat Utilization of Juvenile Atlantic Bluefin Tuna, Thunnus thynnus, Tracked with Mini PSAT and Archival Tags" was published in 2012. Journal: PLoS One.

Under current ABFT management, the 50% maturity ogive considered by ICCAT in stock assessment is 4 years and 8 years, for the eastern and western stocks, respectively [53]. Growth curves, however, show similar rates of growth between Eastern and Western stocks [54] and food habits are also similar [47]. Recent genetic, microconstituent and organo-chlorine sampling of juvenile ABFT demonstrate consistently higher contributions of Mediterranean-origin individuals in the western Atlantic [2], [7], [55] than estimates of mixing returned from conventional tagging studies [8], yet timing, mechanism and frequency of trans-Atlantic exchange are better addressed through electronic tagging [3], [56]. Although natal origin of the tagged fish is not yet fully resolved (Dr. Jan McDowell, personal comm.), presumably, genetic analysis will eventually confirm their origins [55]. If the rates of exchange of age 2–5 ABFT are consistent with biomarker studies it is reasonable to assume that adolescent and maturing ABFT of eastern origin may be present in the western fishery. Consequently, tagging studies of age 2–5 ABFT are particularly important in the western Atlantic to determine annual trans-Atlantic exchange rates of juvenile size classes in stock assessments [56]–[58].

None of the individuals tagged with PSATs in 2007 crossed the 45° deg W management line while monitored, although one fish had a distinct easterly heading when its tag prematurely released (Fig. 1). Although to date there are no known archival tag recoveries from eastern-origin juveniles in the Gulf of Maine, recreational fishermen have recaptured two juveniles released with conventional tags in the Bay of Biscay (76 cm FL) and off Gibraltar (67 cm FL,), respectively, that had been at large for 2–3 years. These fish were about 1–2 years old at release, and when recaptured off Cape Cod, MA, were located in the same area at the same time as fish tagged with PSATs in this study, confirming mixed stocks on western feeding grounds.

Conventional and electronic tagging provide only snapshots of the population as a whole. Some juvenile ABFT cross the Atlantic at age 2, although it is not known whether transits occur annually or whether climatological and/or prey cycles drive them [6], [59]. Although none of the electronically tagged fish crossed the Atlantic during the observation period, biomarkers and conventional tagging suggest the possibility that we tagged eastern-origin fish. Assuming spawning site fidelity, and age of maturity at 3–5 years [60], eastern origin fish located on western forage grounds would presumably return to spawn. If continued on an annual basis over a range of juvenile size classes, electronic tagging could eventually confirm the timing and size of ABFT returning from the western Atlantic to the Mediterranean Sea.

The article "Dispersal Routes and Habitat Utilization of Juvenile Atlantic Bluefin Tuna, Thunnus thynnus, Tracked with Mini PSAT and Archival Tags" was published in 2012. Journal: PLoS One.

Since spatial distributions were generally coincident with recreational fisheries, at present the recreational fleet catch is fairly representative of the overall juvenile bluefin assemblage in summer and fall. Spatial variability, of course, exists in our results and core use areas often appear to be along the shelf break. This could shift the reliability of catch representation since the effective fishing range of typical recreational vessels is usually limited to ∼50 miles from shore. The observed spatial range compression in summer months is an advantage in that it appears to accurately represent the extent of juvenile distribution in that quarter, and based on diet studies, suggests association with sand lance (*Ammodytes* sp.), [10], [47] which form schools composed of tens of thousands of individuals along the Northwest Atlantic shelf [61].

Vertical habitat envelopes are useful in gauging water mass inhabitation of pelagic fishes and can indicate vulnerability to various fishing gear [33]. While current ICCAT regulations prohibit commercial fishing for juvenile ABFT in the western Atlantic, the surface oriented behavior in summer months shown in this study provides important spatio-temporal information for designing and implementing direct assessments utilizing aerial survey, sonar, or LIDAR technologies [37], [62], [63]. Detectability is an important bias in any aerial survey [62], [64], and prior knowledge of when observed animals are likely to be visible is a valuable tool for assessing error rates and enhancing the overall success of an aerial survey. The current population status of Atlantic bluefin tuna and other highly migratory species is disputed, and meta analysis [65], [66] or traditional CPUE-based assessments approaches [67], [68], rely on fishery dependent information that may not match real distribution and abundance [69], [70]. Providing more realistic and timely indices of recruitment for juvenile size classes of ABFT is considered to be one of the highest priorities for future ICCAT stock assessment [54]. Here, we provide evidence that the spatial distributions of juvenile ABFT during the summer and early autumn are within current technical capability for generating a fishery-independent, direct assessment index off the eastern coast of the U.S leading to a better understanding of regional biomass.
